# Clinical Efficacy of Glucosamine plus Sodium Hyaluronate for Osteoporosis Complicated by Knee Osteoarthritis and Its Influence on Joint Function and Bone Metabolic Markers

**DOI:** 10.1155/2022/6078254

**Published:** 2022-08-30

**Authors:** Jing-Jin Yang, Xiu-Mei Zhang

**Affiliations:** ^1^Department of Endocrinology, The First People's Hospital of Huaihua, Huaihua, 418000 Hunan, China; ^2^Department of Gastroenterology, The First People's Hospital of Huaihua, Huaihua, 418000 Hunan, China

## Abstract

**Background:**

Osteoporosis (OP) associated with knee osteoarthritis (KOA) is common in older men and postmenopausal women, and it is important to find reliable and effective treatments for this disease to improve joint function and bone metabolism in this population.

**Objective:**

To clarify the clinical efficacy of glucosamine (GlcN) plus sodium hyaluronate (SH) for OP complicated by KOA (OP + KOA) and its influence on joint function and bone metabolic markers (BMMs).

**Methods:**

Admitted from July 2019 to July 2021, 126 patients with OP + KOA were selected, including 76 cases (observation group) treated with GlcN plus SH and 50 cases (control group) given GlcN alone. The pain, joint function, BMMs, and clinical efficacy were evaluated and compared. Pain and joint function assessments employed the Visual Analogue Scale (VAS) and the Western Ontario and McMaster Universities Osteoarthritis Index (WOMAC) plus Lysholm Knee Scoring Scale, respectively. BMMs mainly measured bone gla protein (BGP), serum tartrate-resistant acid phosphatase variant (TRACP)-5b, type I collagen cross-linked C-telopeptide (CTX-1), and bone-specific alkaline phosphatase (BALP).

**Results:**

Higher posttreatment VAS scores were determined in observation group as compared to control group; observation group showed lower WOMAC scores of joint function and higher Lysholm scores than control group; in terms of BMMs, TRACP-5b and CTX-1 were lower while BGP and BALP were higher in observation group; the curative effect was also higher in observation group. All the above differences were statistically significant.

**Conclusions:**

GlcN plus SH has definite clinical efficacy in the treatment of OP + KOA, which can not only significantly improve patients' joint function and bone metabolism but also relieve pain, with high clinical popularization value.

## 1. Introduction

Osteoporosis (OP), a metabolic bone disease characterized by reduction of bone per unit volume and bone microstructure degeneration, has a predilection for elderly men and postmenopausal women and is associated with bone pain and fractures [1]. Knee osteoarthritis (KOA) is a degenerative joint disease in which articular cartilage is destroyed, and subchondral bone is hardened [2]. With the influence of bone degeneration factors, most patients will develop KOA accompanied by OP [3]. This is also related to the fact that the two diseases have common pathogenic factors such as gender, heredity, and inflammation [4]. Patients with OP complicated by knee KOA (OP + KOA) will experience symptoms such as pain and limited activity, which not only affects their quality of life but also imposes certain burdens on their families and social economy [5]. At present, the treatment options for these diseases are mainly a balanced diet, calcium and vitamin D supplementation, exercise, and other lifestyle measures, as well as drug treatments such as bisphosphonates and teriparatide. The above nondrug treatment methods are challenging for patients, difficult to adhere to and slow to respond, while bisphosphonate, telipatide, and other drug therapies have toxic side effects with contraindications in some patients [6]. Therefore, it is particularly important to find an effective method to treat OP + KOA.

Glucosamine (GlcN), a natural amino monosaccharide, is the precursor of proteoglycan synthesis and is used in various types of arthritis [7], effectively stimulating chondrocyte synthesis [8]. It has been shown to effectively inhibit granulation growth and vascular exudation in the treatment of osteoarthritis, thus inhibiting delayed allergic reaction [9]. Intra-articular injection of sodium hyaluronate (SH) is a common clinical treatment for OP + KOA [10]. SH is a component of synovial fluid and articular cartilage, which can improve the mechanical lubrication of joints. In addition, it can rebuild and repair the damaged physiological barrier, reduce articular cartilage friction-induced pain, improve joint mobility, and relieve patients' clinical symptoms [11]. Evidence has shown that the effective components of SH injection can also combine with glycoproteins in synovial fluid, thus blocking the inflammatory reaction process and effectively improving patients' diseases [12]. However, there are few studies reporting the application of GlcN plus SH in the treatment of OP + KOA. Consequently, we tested a series of indicators such as bone metabolic markers (BMMs) and joint function, to examine the efficacy of the combined treatment for the disease.

## 2. Data and Methods

### 2.1. General Case Data

This study retrospectively enrolled 126 OP + KOA patients admitted from July 2019 to July 2021, including 76 patients (observation group) treated with GlcN plus SH and 50 patients (control group) intervened by GlcN alone. This study was approved by the Academic Ethics Committee of The First People's Hospital of Huaihua. All patients participating in this study were fully aware of the purpose of this study and signed informed consent. All the enrolled cases were diagnosed as OP + KOA by X-ray plain film or CT examination [13], independent of alcohol and drugs, and could correctly understand the relevant contents of the scales used and answer the questions, with the Kellgren-Lawrence (K-L) grade I or II [14], complete general clinical data, and no recent use of other related therapeutic drugs, while those who had received knee joint replacement, with severe mental disorders, allergies to the study medication, and noncompliance with the research were excluded, as well as withdrawals and loss to follow-ups.

### 2.2. Therapeutic Methods

Both groups received basic treatment, including inflammatory and pain interventions. Patients in control group were treated with GlcN (Kangbide Pharmaceutical, Beijing, China, H20070173), 0.72 g each time, twice daily, for 5 weeks. On this basis, observation group was given SH injection (Bausch & Lamb Freda Pharmaceutical, Shandong, China, H10960136) once a week, 25 mg each time, also for 5 weeks.

### 2.3. Blood Sampling

Before and 5 weeks after treatment, 5 mL of fasting venous blood was drawn from patients in both groups at 8 am and sent to the laboratory for centrifugation, and the resulting supernatant was stored into anticoagulant tubes. All serum samples were used within 6 h.

### 2.4. Endpoints

1. Visual Analogue Scale (VAS) score [15]: patients' pain degrees were assessed before and after treatment with the VAS, an instrument with a score ranging from 0 (painless) to 10 points (unbearable pain). Higher scores indicate greater pain severity
2. The joint function score was evaluated by the Western Ontario and McMaster Universities Osteoarthritis Index (WOMAC, score range: 0-96 points) [16] and Lysholm Knee Scoring Scale (score range: 0-100 points) [17]. The former evaluated knee structure and function, including treatment for pain, stiffness, and joint function. A higher score indicates more severe arthritis. With the latter, patients were assessed for support, colic, locking sensation, joint instability, joint swelling, difficulty in stair-climbing, etc. Higher scores represent better recovery
3. Enzyme-linked immunosorbent assays (ELISAs) [18] were also carried out to measure BMMs before and after treatment: the tests were carried out strictly according to the instructions of human BGP, TRACP-5b, CTX-1, and BALP ELISA kits (Shanghai Yuanmu Biotech, Cat. Nos. YM-S0840, YM-SZ0827, YE00708, YM-SZ0822)
4. Efficacy evaluation: it was considered a marked response if there was significant relief in lower back and knee joint pain, with restored knee joint activity function; response was defined as alleviated lower back and knee pain compared with before treatment, with improved knee joint motion function; and nonimprovement in the patient's symptoms with aggravated pain after treatment is regarded as nonresponse. overall response rate (ORR) = (marked response + response) cases/total cases × 100%

In this study, VAS score, WOMAC score, and Lysholm score were secondary endpoints, while BGP, TRACP-5b, CTX-1, BALP, and efficacy were primary endpoints.

### 2.5. Statistical Methods

Data statistical analysis and visualization adopted SPSS21.0 (SPSS, Inc., Chicago, IL, USA) and GraphPad Prism 6.0 software (GraphPad Software Inc., San Diego, CA, USA), respectively. The method for within-group comparisons of counting data recorded as the number of cases/percentage [*n* (%)] was the chi-square test, or chi-square continuity correction when the theoretical frequency of the former test was under 5. The mean ± SD was used to indicate measurement data; for measurement data analysis, independent samples *t*-test was used for between-group comparisons, while paired *t*-test was used for within-group ones. The threshold of significance was *P* < 0.05 in this research.

## 3. Results

### 3.1. General Information

As shown in Table 1, the two cohorts of patients were nonsignificantly different in mean age, average course of disease, body mass index, smoking history, drinking history, hypertension history, K-L grading, and other general clinical baseline data (*P* > 0.05).

### 3.2. Comparison of Pre- and Posttreatment VAS Scores

No statistical difference was observed in the pre-treatment VAS score between control group and observation group (*P* > 0.05), but after treatment, the VAS score of the two groups was significantly improved, with a markedly lower score in observation group (*P* < 0.05) (Figure 1).

### 3.3. Comparison of Pre- and Posttreatment Joint Function Scores

No statistical differences were found in pretreatment WOMAC and Lysholm scores between observation group and control group (*P* > 0.05). After treatment, both the WOMAC and Lysholm scores changed significantly in the two groups, with a lower WOMAC score and a higher Lysholm score in observation group compared with control group (*P* < 0.05) (Figure 2).

### 3.4. Comparison of Pre- and Posttreatment BMMs

The BMMs (BGP, TRACP-5b, CTX-1, and BALP) differed insignificantly between groups prior to treatment (*P* > 0.05). After treatment, BGP, TRACP-5b, CTX-1, and BALP of the two groups were significantly improved, with statistically lower TRACP-5b and CTX-1 while higher BGP and BALP in observation group as compared to control group (Figure 3).

### 3.5. Comparison of Clinical Efficacy after Treatment

After treatment, the ORR was found to be 93.42% in observation group and 78.00% in control group, with statistical significance (*P* < 0.05) (Table 2).

## 4. Discussion

In OP + KOA patients, the damaged articular surface will be in a state of long-term friction, which would induce a large number of wear particles and stimulation of synovial nociceptors, causing joint osteoarthritis [19]. The capsular cavity of the knee joint is abundant in blood vessels and nerves. If there is joint trauma, the synovium and ligament in the joint will be congested, and massive inflammatory exudate will be released, which will affect the knee joint function of patients [20]. At present, various treatments are available for the disease, but all with unsatisfactory curative effects [21]. Hence, this study is to observe the effect of GlcN plus SH on this disease, aiming to find a better alternative for the disease.

GlcN can effectively promote the production of glycosaminoglycans and proteoglycans to promote the synthesis of knee cartilage, with some certain anti-inflammatory effects [22], while SH can actively participate in the regulation of electrolyte and water in the extracellular fluid after entering the patient's body, which can validly lubricate joints, resist infection and heal wounds, and effectively lubricate joint cavities, thus protecting joints [23]. In the research of Wang et al. [24], SH plus GlcN for KOA patients effectively mitigated joint pain, promoted the functional recovery of knee joints, and enhanced the therapeutic effect. Alekseeva et al. [25] reported that hyaluronic acid plus chondroitin sulfate and glucosamine hydrochloride can effectively improve patients' life quality and reduce joint pain. Our study results revealed a statistically lower VAS score in observation group compared with control group after treatment. It indicates that GlcN plus SH can effectively promote articular cartilage synthesis, eliminate inflammation caused by OP + KOA, and play the role of cartilage preservation, thus effectively relieving pain. In the study of Brandt et al. [26], SH significantly reduced knee pain and stiffness of KOA patients, improved their joint function, and provided lasting benefits for those with moderate knee pain. And according to Muraleva et al. [27], the administration of GlcN to an animal model of OP reduced bone loss. In terms of joint function, our study identified that the WOMAC score was significantly lower while the Lysholm score was higher in observation group as compared to control group, demonstrating that GlcN plus SH can not only effectively relieve the pain symptoms and swelling of patients but also effectively improve their joint mobility.

Biomarkers of bone turnover can be used as a better way than radiographs to observe osteoarthritis progression [28]. BGP and BALP, as markers of bone formation, and TRACP-5b and CTX-1, as markers of bone resorption, can effectively reflect changes in bone metabolism in patients and indirectly reflect alterations in joint function [29, 30]. Our findings identified statistically lower BMMs TRACP-5b and CTX-1 while higher BGP and BALP in observation group after treatment. It indicates that after the combined treatment of GlcN and SH, bone absorption decreases, and bone formation begins to increase, which effectively corrects the imbalance of bone metabolism. It also shows that the combination therapy can effectively realize fracture healing and improve bone structure. Moreover, the curative effect was obviously higher in observation group versus control group, suggesting that GlcN plus SH has a definite clinical effect in treating OP + KOA, which can effectively reduce pain, improve knee joints, and promote rapid recovery from the disease.

Although this work has confirmed that GlcN plus SH is effective for OP + KOA, there is still some deficiencies and room for improvement. For example, we can supplement basic experiments on the therapeutic mechanisms of the two treatments to explore the risk factors that influence patient outcomes at the molecular level. Second, the sample size can be increased to improve the accuracy of experimental results. Third, prognostic analysis should be supplemented to further understand the effect of GlcN plus SH on the prognosis of such patients. We will gradually improve the research from the above perspective in the future. In addition, the innovation of this study is to compare and analyze the clinical effects of GlcN plus SH and GlcN monotherapy in the treatment of OP + KOA in terms of pain, joint function, BMMs, clinical efficacy, etc., which confirms the clinical effectiveness of the combination therapy and provides a new direction and reliable basis for the treatment of such patients.

## 5. Conclusion

Taken together, GlcN plus SH is superior to GlcN monotherapy for patients with OP + KOA, which can not only significantly relieve pain, improve patients' joint function and bone metabolism but also further improve the curative effect, with high clinical promotion value.

## Figures and Tables

**Figure 1:** Comparison of pre- and posttreatment VAS scores. The VAS score was not statistically different between groups before treatment, but the score was significantly lower in the observation group compared with the control group after treatment. Note: ^∗^ indicates *P* < 0.05 compared with before treatment or between two groups.

**Figure 2:** Comparison of pre- and posttreatment joint function scores. (a) The WOMAC score of the observation group was not statistically different from that of the control group before treatment, but after treatment, the score was statistically lower in the observation group. (b) The Lysholm score of the observation group was not statistically different from that of the control group before treatment, but the score was statistically higher in the observation group after treatment. Note: ^∗^ indicates *P* < 0.05 compared with before treatment or between two groups.

**Figure 3:** Comparison of pre- and posttreatment bone metabolism indexes. (a) The BGP of the observation group was not statistically different from that of the control group before treatment, but after treatment, the BGP was statistically higher in the observation group. (b) The TRACP-5b of the observation group was not statistically different from that of the control group before treatment, but it was statistically lower in the observation group after treatment. (c) The CTX-1 of the observation group was not statistically different from that of the control group before treatment, but after treatment, it was statistically lower in the observation group. (d) The BALP of the observation group was not statistically different from that of the control group before treatment, but it was statistically higher in the observation group after treatment. Note: ^∗^ indicates *P* < 0.05 compared with before treatment or between two groups.

**Table 1:** Comparison of general data [*n* (%)] (mean ± SD).

Classification	Observation group (*n* = 76)	Control group (*n* = 50)	*t*/*χ*^2^	*P*
Average age (years old)	52.07 ± 5.07	53.14 ± 5.39	1.130	0.261
Average course of disease (years)	3.80 ± 1.41	3.56 ± 1.55	0.898	0.371
Body mass index (kg/m^2^)	24.70 ± 2.54	24.04 ± 2.11	1.523	0.130
Smoking history			2.119	0.145
Yes	45 (59.21)	23 (46.00)		
No	31 (40.79)	27 (54.00)		
Drinking history			0.007	0.935
Yes	42 (55.26)	28 (56.00)		
No	34 (44.74)	22 (44.00)		
History of hypertension			0.132	0.716
Yes	37 (48.68)	26 (52.00)		
No	39 (51.32)	24 (48.00)		
K-L grading			0.366	0.545
I	43 (56.58)	31 (62.00)		
II	33 (43.42)	19 (38.00)		

**Table 2:** Comparison of clinical efficacy after treatment [*n* (%)].

Groups	Marked response	Response	Nonresponse	Overall response rate (%)
Observation group (*n* = 76)	48 (63.16)	23 (30.26)	5 (6.58)	71 (93.42)
Control group (*n* = 50)	17 (34.00)	22 (44.00)	11 (22.00)	39 (78.00)
*χ* ^2^	—	—	—	6.469
*P*	—	—	—	0.011

## Data Availability

The labeled dataset used to support the findings of this study are available from the corresponding author upon request.
